The article "Do Higher Education and Financial Institutions Improve Health in China? A New Perspective" was retracted in 2025. Reasons: an official misconduct investigation; compromised peer review; a compromised editor; unreliable results or conclusions.

# Do Higher Education and Financial Institutions Improve Health in China? A New Perspective

**DOI:** 10.3389/fpubh.2022.874507

**Published:** 2022-03-18

**Authors:** Zhan Zhan, Ran Tao, Muhammad Umer Niaz, Dervis Kirikkaleli

**Affiliations:** ^1^School of Business, Wuchang University of Technology, Wuhan, China; ^2^Qingdao Municipal Center for Disease Control and Prevention, Qingdao, China; ^3^Faculty of Management and Social Sciences, Capital University of Science and Technology (CUST), Islamabad, Pakistan; ^4^European University of Lefke, Faculty of Economic and Administrative Science, Department of Banking and Finance, Lefke, Turkey

**Keywords:** higher education, financial institutions, health, China, ARDL

## Abstract

The importance of human wellbeing is documented in the literature of development economics because of its intensifying impacts on economic growth and productivity of labor in the long-run. To the best of the authors' knowledge, no empirical study has examined the symmetric association between China's financial institutional development, education, and health outcomes. Thus, our study aims to fill this vacuum by employing an autoregressive distributed lag (ARDL) approach to explore the impact of financial institutional development and education on life expectancy and infant mortality rate from 1990 to 2020. The empirical analysis reveals that financial institutional development and education report a significant increase in life expectancy and meaningful reduction in mortality rate in the long-run. Based on these findings, the study may deliver intuitive policy implications regarding improvement in health conditions that are imperative for promoting economic growth in the long-run.

## Introduction

In view of the welfare economists, the contribution of income development is the key determinant to the satisfaction of households (1). Consequently, Di Tella et al. (2) denoted that income increases only provide temporary satisfaction to individuals. For example, Veenhoven (3) study reported that the increase in income no longer affects the happiness of households, revealing that income affects happiness only until the necessities are fulfilled. After that point increase in income empowers people to avail themselves of health facilities for themselves and their children. Resultantly, improvement in the happiness of households came from the decline in infant and child mortality. Ebenstein et al. (4) reported that millions of children were decimated due to intense poverty, lack of basic needs, malnutrition, and lack of access to public health. In contrast, Easterlin (5) denoted that the happiness of individuals is not linked with an increase in per capita income. The study added that there is no long-run association between the incomes of the nation and the satisfaction level of people (6). However, improvement in satisfaction level of people depends on the health and other family circumstances such as marital status and employment. Additionally, Kahneman (7) claimed the fundamental factors of life satisfaction nullify the impacts of income level.

The article "Do Higher Education and Financial Institutions Improve Health in China? A New Perspective" was retracted in 2025. Reasons: an official misconduct investigation; compromised peer review; a compromised editor; unreliable results or conclusions.

Kahneman and Deaton (8) argued that the high-income level only enhances the life evaluation but not the emotional welfare. Likewise, the Human Development Report of UNDP (1990) highlighted that the leading determinants of human development are decent living, adult literacy, life expectancy, and reduction in mortality rate. Among all determinants of human development, reduction in mortality rate and life expectancy are the fundamental sources of human wellbeing (1). Sen (9) denoted that easy access to social services such as sanitation, health care, better provision of education, and clean water for drinking leads to improvement in human development thus, improving life expectancy and reducing the mortality rate (10). Hence, it can be claimed that the proficiency development of social services is the key source of healthy life expectancy. Given the significance of both the income approach and capability approach, it is still disappointing that the developing economies present high mortality rates and poor life expectancy in this era of globalization (11). Thus, it has become a dire need of time to understand the key determinants of healthy life expectancy on several grounds.

In literature, education is considered a key determinant of health. It is argued that a persistent and large association exists between health and education. The nexus between health and education has been measured in various economies for different time periods, including various health measures. In literature, considerable attention has been given to health inequalities. Economies have settled their health goals. For instance, the United Kingdom has set the goal of reducing health-related disparities through educational support. The positive linkage between health and education is well constructed theoretically and empirically. Educated households experience good health compared to less educated as shown by their self-reported good physical health and functioning, lower mortality rates, morbidity, and disability. However, less education is attached to a high prevalence of chronic diseases, infectious diseases, short life expectancy, and poor health and functioning (12–14). Education improves health outcomes and improves abilities of thinking and decision-making (15). Popay et al. (16) denoted that educated people possess better knowledge regarding self-care during chronic diseases, such as using inhalers correctly during asthma conditions.

The article "Do Higher Education and Financial Institutions Improve Health in China? A New Perspective" was retracted in 2025. Reasons: an official misconduct investigation; compromised peer review; a compromised editor; unreliable results or conclusions.

The development of financial institutions is also considered a significant determinant of human development. Claessens and Feijen (17) study revealed that financial development may influence life expectancy through various channels. The first channel is described through the income effect, which states that financial development boosts economic output and industrialization. Economic activity growth and industrialization create employment opportunities and raise income levels (18). The increase in the level of income enables people to save money, afford better food, housing, nutritional intake, health-care facilities, working conditions, better living standards, and thus enhance the overall life expectancy. The second channel is described through the education effect, which reveals that financial development helps people spend more money for higher education that improves their skills for more employment opportunities. With good quality education and a better level of income, people become more conscious about health, which improves their life expectancy. The third channel is described through the effect of gender equality which states that financial development enables women to participate in income-generating activities. Self-employed women can take good care of their children and can spend more income on health. Consequently, financial institutions' development indirectly improves life expectancy and family health. Finally, the fourth channel is described through the infrastructure effect. Infrastructure development enhances economic growth via both private and public investments in building infrastructure for health care such as clinics, hospitals, and the availability of medicines (19).

In literature, very limited studies have analyzed the impact of education and the development of financial institutions on health outcomes. To fill this vacuum, this research contributes to the existing stock of literature by being the pioneer study to examine the impact of education and financial institutional development on health outcomes in China. The study adopted the Autoregressive Distributed Lag (ARDL) approach for conducting empirical inferences from 1990 to 2020. The study has also theoretical and empirical contributions to the literature. This study employs ARDL to explore the long and short-run effects of higher education and financial institutions on human health. The findings of this study will provide intuitive policy implications for improvement in health outcomes through financial institutional development and education. Both determinants are of crucial importance for enhancing life expectancy in China.

The article "Do Higher Education and Financial Institutions Improve Health in China? A New Perspective" was retracted in 2025. Reasons: an official misconduct investigation; compromised peer review; a compromised editor; unreliable results or conclusions.

## Model and Methods

The theoretical and empirical literature has proposed that education is vital for health outcomes. Education plays an important role in increasing the stock of human capital and improving the quality of life. The financial institution's development also has a favorable impact on health outcomes through income and skills channels. Internet improves health via knowledge, self-awareness, e-health, and digital inclusion. FDI also positively impacts the quality of life (20, 21). A time series model is used and written as:


(1) $$\begin{array}{l} \;\begin{array}{c} Health_{\;t}=\;\lambda_{0}+\lambda_{1}HE_{t}+\lambda_{2}FID_{t} \end{array}\\ \begin{array}{c} +\lambda_{3}GDP_{t}+\lambda_{4}Internet_{t}+\lambda_{5}FDI_{t}+\varepsilon_{t} \end{array} \end{array}$$

Where Health is health outcomes, HE is higher education, FID signifies financial institutions development, GDP per capita specifies the economic performance, the Internet is the internet users, and FDI is foreign direct investment. Education provides awareness and information of health, thus λ_1_ will be positive. Financial institutions development can also improve clean fuels and technologies by reducing the financial constraints, thus an estimate of λ_3_ to be negative. Finally, the internet and FDI boost health; thus, estimate of λ_4_ & λ_5_ will be positive. The basic model has presented only long-run parameter estimates. We prolong our basic model into an error-correction format by obtaining short-run parameter estimates as follows:


(2) $$\begin{array}{l} \begin{array}{c} \text{ Δ}Health_{t}=\;\varphi_{0}+\;\sum_{k=1}^{n}\alpha_{1k}\text{Δ}Health_{\;t-k}\\ \;+\;\sum_{k=0}^{n}\alpha_{2k}\text{Δ}HE_{\;t-k}+\sum_{k=1}^{n}\alpha_{3k}\text{Δ}FID_{\;t-k}\\ \;+\sum_{k=0}^{n}\alpha_{4k}\text{Δ}GDP_{\;t-k}+\sum_{k=1}^{n}\alpha_{5k}\text{Δ}Internet_{\;t-k}\\ \;+\;\sum_{k=0}^{n}\alpha_{6k}\text{Δ}FDI_{\;t-k}+\;\lambda_{1}Health_{\;t-1}+\;\lambda_{2}HE_{t-1}+\lambda_{3}FID_{\;t-1} \end{array}\\ \begin{array}{c} +\;\lambda_{4}GDP_{\;t-1}+\lambda_{5}Internet_{\;t-1}+\;\lambda_{6}FDI_{\;t-1}+\lambda .\;ECM_{\;t-1}+\varepsilon_{t} \end{array} \end{array}$$

Specification (2) now resembles the autoregressive distributive lag order (ARDL) model of Pesaran et al. (22). The ARDL is considered superior as compared to other time series models in many aspects. For instance, in other time series techniques it is mandatory to check the stationarity of the variables and the variables must be integrated at the same order (23). However, in the ARDL model Pre-unit root testing is not mandatory because it can account for integrating properties of the variables and can also analyze the variables whether they are stationary at level or at first difference. Another benefit of this method is that it can provide both short and long simultaneously. In the above equation (2) the short-run estimates are those that are attached to the first difference variables and the long-run estimates are connected to coefficients π_2_−π_6_ normalized on π_1_. However, these long-run estimates are considered valid only if they are cointegrated. To that end, Pesaran et al. (24) proposed an F-test for the joint significance of the lagged level variables and also developed critical values for this test. If the calculated value of the *F*-test is greater than the critical values this is confirmation of valid long-run results. Another important benefit of this method is that it performs well even if the sample size is small (25). Lastly, this method also includes a short-run dynamic process, which helps to analyze any feedback effect, which is crucial for removing multicollinearity and endogeneity (26).

The article "Do Higher Education and Financial Institutions Improve Health in China? A New Perspective" was retracted in 2025. Reasons: an official misconduct investigation; compromised peer review; a compromised editor; unreliable results or conclusions.

## Data

The study investigates the impact of higher education and the development of financial institutions on health outcomes in China. The study uses data for the period 1991 to 2020 for empirical investigation. Definitions, descriptions of data, and statistical inferences are given in Table 1. Health outcome is measured by life expectancy (in total years) and mortality rate (per 1,000 live births). Higher education is measured as tertiary education level. However, the role of financial institutions is measured as the development of financial institutions. Besides these variables, GDP, internet, ICT, FDI, and patent are used as control variables. Where GDP is taken at constant 2015 US$, the internet is measured by total internet users as a percent of the total population, ICT is measured by ICT index, net inflows as a percent of GDP are taken to measure FDI, and patent is measured by total residents and Non-residents patent applications. The required data have been extracted from the World Bank and IMF.

**Table 1:** Definitions and descriptions.

**Variables**	**Definitions**	**Mean**	**Std. Dev**.	**Min**	**Max**
IM	Mortality rate, infant (per 1,000 live births)	21.78	12.34	1.639	41.70
LE	Life expectancy at birth, total (years)	73.08	2.571	69.24	77.31
HEDU	School enrollment, tertiary (% gross)	22.15	17.68	2.806	58.42
FIE	Financial institutions development	0.750	0.040	0.648	0.799
GDP	GDP per capita (constant 2015 US$)	8.187	0.750	6.883	9.420
Internet	Individuals using the Internet (% of population)	22.36	24.00	0.000	70.64
ICT	ICT index	26.32	25.09	0.152	73.56
FDI	Foreign direct investment, net inflows (% of GDP)	3.389	1.341	1.139	6.187
Patent	Patent applications, total (residents and Non-residents)	12.02	1.667	9.343	14.75

The article "Do Higher Education and Financial Institutions Improve Health in China? A New Perspective" was retracted in 2025. Reasons: an official misconduct investigation; compromised peer review; a compromised editor; unreliable results or conclusions.

## Results and Discussion

The study employed the Phillips Perron (PP), and Dickey-Fuller Generalized Least Square (DF-GLS) tests to detect unit-root properties. The findings of both unit root tests are given in Table 2. The PP test observed that the development of financial institutions (FIE) and foreign direct investment (FDI) are level stationary variables while the remaining are first difference stationary variables. In the case of the GF-GLS test, it is observed that the development of financial institutions (FIE), ICT, and foreign direct investment (FDI) are level stationary variables and the rest are first difference stationary variables. Based on the findings of both unit root tests, our study applied the ARDL approach for empirical testing of the long-run association between variables. Table 3 reports the long-run and short-run findings of ARDL models. So far, our study has measured health outcomes in China through two proxies, i.e., infant mortality and life expectancy. Thus, we have regressed two separate ARDL models.

**Table 2:** Unit root tests.

	**PP**			**DF-GLS**		
	**I(0)**	**I(1)**	**Decision**	**I(0)**	**I(1)**	**Decision**
IM	−0.128	−3.202^**^	I(1)	0.988	−1.966^**^	I(1)
LE	0.214	−2.678^*^	I(1)	0.235	−1.689^*^	I(1)
HE	1.230	−2.658^*^	I(1)	0.254	−2.653^***^	I(1)
FIE	−3.102^**^		I(0)	−1.867^*^		I(0)
GDP	−0.875	−3.210^**^	I(1)	0.212	−1.852^*^	I(1)
Internet	1.255	−2.657^*^	I(1)	0.120	−1.652^*^	I(1)
ICT	1.652	−2.675^*^	I(1)	−1.925^**^		I(0)
FDI	−2.758^*^		I(0)	−1.765^*^		I(0)
Patent	0.235	−9.025^***^	I(1)	0.325	−5.265^***^	I(1)

* *p < 0.1*,

** *p < 0.05*,

*** *p < 0.01*.

**Table 3:** ARDL estimates of human health.

	**IM**		**LE**	
**Variable**	**Coefficient**	***t*** **-Stat**	**Coefficient**	***t*** **-Stat**
**Short-run**				
HEDU	−0.022^*^	1.745	0.102^*^	1.827
HEDU (−1)	0.027	0.527	−0.002	0.802
HEDU (−2)	0.039	1.126	0.003^*^	1.923
FIE	−0.354	1.369	0.284^*^	1.680
GDP	−2.742^***^	12.25	1.590^***^	16.34
GDP (−1)	0.510^***^	7.680	−1.431^***^	13.70
Internet	0.034	1.088	0.005^***^	5.430
FDI	0.356^**^	2.365	−0.013^**^	2.420
FDI (−1)	0.096	1.151		
FDI (−2)	0.149	1.625		
**Long-run**				
HEDU	−0.085^**^	2.235	0.028^***^	3.544
FIE	−1.037	1.568	2.209^*^	1.788
GDP	−1.962^***^	11.83	1.235^***^	2.845
Internet	−0.066	1.173	0.039^***^	4.058
FDI	1.170^***^	3.193	−0.099^**^	2.195
C	4.206^***^	18.26	7.950^***^	26.53
**Diagnostics**				
*F*-test	21.02^***^		6.654^***^	
ECM (−1)^*^	−0.513^***^	14.36	−0.428^***^	15.77
LM	1.356		0.345	
BP	0.332		0.254	
RESET	0.247		0.147	
CUSUM	S		S	
CUSUM-sq	S		S	

* *p < 0.1*,

** *p < 0.05*,

*** *p < 0.01*.

The article "Do Higher Education and Financial Institutions Improve Health in China? A New Perspective" was retracted in 2025. Reasons: an official misconduct investigation; compromised peer review; a compromised editor; unreliable results or conclusions.

In the Infant mortality model, the long-run findings display a negative association between higher education and infant mortality rate describing that due to an increase in the level of education, the infant mortality rate reduces significantly. The coefficient estimates display that a 1 percent increase in the level of education declines the infant mortality rate by 0.085 percent in the long-run. In contrast, the development of financial institutions reports an insignificant impact on the infant mortality rate in the long-run. The findings of control variables display that GDP is negatively associated with infant mortality rate revealing that a 1 percent escalation in GDP brings a 1.962 percent reduction in infant mortality rate in the long-run. However, the internet reports an insignificant impact on infant mortality rate in the long-run. The long-run findings demonstrate a positive linkage between FDI and infant mortality rate, inferring that a 1 percent increase in FDI inflow causes a 1.170 percent increase in infant mortality rate in China. In the short-run, the findings report that higher education brings a significant reduction in infant mortality rate while the development of financial institutions reports an insignificant impact on infant mortality rate. In the short-run, GDP brings a significant reduction in infant mortality rate while FDI brings significant increases in infant mortality rate. Again, the internet reports no significant impact on infant mortality rate in the short-run.

In the life expectancy model, the long-run findings reveal that higher education is positively associated with life expectancy, confirming that life expectancy increases significantly due to an upsurge in the level of education. The coefficient estimate reports that a 1 percent increase in the level of education increases life expectancy by 0.028 percent in the long-run. Education directly causes health by affecting human behaviors, and this empirical finding is also supported by (27). This also means that education positively affects human health by improving social development. Education improves human health and wellbeing by reducing poverty and income inequality. The positive effects of higher education on human health by improving income level, skills, and financial development this finding are also supported by (28). Education is an important contributor to health by improving technical changes in the economy.

The long-run findings reveal a positive association between the development of financial institutions and life expectancy, which shows that a 1 percent upsurge in the development of financial institutions tends to increase life expectancy by 2.209 percent. The finding is in line with Shahbaz et al. (19), who noted that financial institutions' development is more likely to improve life expectancy by reducing infant mortality rate and increasing life expectancy through education, income, wealth, gender equality, infrastructure, and technology affects. Our finding is also backed by Stubbs et al. (29), who noted that International financial institutions positively affect public health. The finding is also backed by Singh & Yadava (30), who noted that financial institutions increase human development. This is expected as small increases in financial institutions' development could potentially promote health by financing health insurance, providing loans, and clinical care. A similar finding is also reported by Pronyk et al. (31), who found that microfinance institutions expanded their services in developing economies and provided health insurance and health education.

The article "Do Higher Education and Financial Institutions Improve Health in China? A New Perspective" was retracted in 2025. Reasons: an official misconduct investigation; compromised peer review; a compromised editor; unreliable results or conclusions.

GDP and life expectancy are positively linked, as shown by the coefficient estimate, which demonstrates that 1 percent intensification in GDP increases life expectancy by 1.235 percent in the long-run. Internet reports a positive impact on life expectancy in the long-run, which states that a 1 percent increase in the use of the internet improves life expectancy by 0.039 percent in the long-run. In contrast, findings display the negative impact of FDI on life expectancy, revealing that a 1 percent increase in FDI inflow reduces life expectancy by 0.099 percent in the long-run. The short-run findings of the model report significant and positive impact of higher education and development of financial institutions on life expectancy, confirming that in response to an increase in the level of education and development of financial institutions, life expectancy improves. In the case of control variables, short-run findings report the positive impact of GDP and the internet on life expectancy and the negative impact of FDI on life expectancy. The robustness of the findings has been confirmed by employing a variable-based method. The findings of the robust models are given in Table 3. Instead of internet and FDI, ICT and Patent variables are used in regressions. In robust models in Table 4, the short-run and long-run findings are quite similar to the findings of actual models.

**Table 4:** ARDL estimates of human health (Robustness).

	**IM**		**LE**	
**Variable**	**Coefficient**	***t*** **-Statistic**	**Coefficient**	***t*** **-Statistic**
**Short-run**				
HEDU	−0.044	1.554	0.013	0.267
FIE	−0.837	0.172	0.025^**^	2.113
FIE (−1)	0.985	1.240	0.378^**^	2.329
FIE (−2)	0.072	1.247	0.310^**^	2.569
GDP	−1.134^***^	8.733	1.450^***^	9.654
GDP (−1)	1.166^***^	6.052	−1.603^***^	5.738
GDP (−2)			0.493^*^	1.678
ICT	0.027	0.476	0.024^**^	2.416
ICT (−1)	−0.183	1.537		
ICT (−2)	0.268	3.779		
Patent	−1.345^***^	2.975	0.032	1.261
**Long-run**				
HEDU	−0.101^*^	1.818	0.032^**^	2.261
FIE	−1.009	0.846	1.786^***^	2.623
GDP	−1.294^***^	5.833	2.281^***^	6.278
ICT	−0.261^***^	6.249	0.026^**^	2.102
Patent	−2.130^***^	3.214	0.212	1.343
C	7.842^***^	13.36	4.139^***^	23.24
**Diagnostics**				
*F*-test	13.21^***^		12.25^***^	
ECM (−1)^*^	−0.430^***^	11.31	−0.549^***^	10.81
LM	1.452		0.332	
BP	1.254		1.254	
RESET	0.687		1.874	
CUSUM	S		S	
CUSUM-sq	S		S	

* *p < 0.1*,

** *p < 0.05*,

*** *p < 0.01*.

The article "Do Higher Education and Financial Institutions Improve Health in China? A New Perspective" was retracted in 2025. Reasons: an official misconduct investigation; compromised peer review; a compromised editor; unreliable results or conclusions.

The findings of F-statistics reveal that a long-run cointegration relationship exists among variables in all the models. The ECM terms are negative and significant in all the models confirming the convergence toward stability. The LM and BP test findings confirm that there is no heteroskedasticity and autocorrelation in the models. The findings of the Ramsey RESET test confirm the correct specification of models. The CUSUM and CUSUM-sq test output confirms the overall stability of the models.

## Conclusion and Policy Implications

Health does not only mean the absence of disease and disability, but it represents a situation of complete physical, mental, and social wellbeing of the people in the society. As society becomes more affluent, it can invest more in the health facilities such as hospitals, laboratories, diagnostic centers, and blood banks. Human capital is a by-product of education, which can be used as an input in the production function to spur economic growth and make people more aware of their health status. The demand for better health facilities also increases in an educated society. Similarly, on one side, the financial institutions can speed up the economic development process that is crucial for better health facilities. On the other side, financial institutions can provide necessary funds to develop health infrastructure. Consistent with this view, our primary focus is to see the impact of education and financial institutions on health in China. We have used two variables to represent health status: infant mortality rate and life expectancy rate.

First of all, we have checked the stationary of the variables via PP and DF-GLS tests, confirming that our variables are a mixture of I(0) and I(1). Therefore, we have employed the ARDL model to estimate the variables. In the long run, the estimated coefficients of higher education turn out to be positive in the case of life expectancy and negative in the case of infant mortality. In the robust model, the long-run estimate of higher education is positive in the context of life expectancy and negative in the case of infant mortality. These results suggest that higher education can benefit both health status indicators, i.e., infant mortality and life expectancy. On the other side, the long-run estimate of financial institutions is positively significant in both the baseline and robust model only in the context of life expectancy, whereas insignificant in the context of infant mortality. These long-run results are valid only if we find co-integration among the long-run variables subject to the significant values of bounds *F*-test or ECM (−1). The estimates of both the tests are significant, confirming the validity of our long-run results. In the short run, higher education and financial institutions prove beneficial for raising people's health status in China.

The article "Do Higher Education and Financial Institutions Improve Health in China? A New Perspective" was retracted in 2025. Reasons: an official misconduct investigation; compromised peer review; a compromised editor; unreliable results or conclusions.

These results help provide policy guidelines. To raise the health status of the people, the government should try to raise the literacy rate in the society because as the people become more educated, they become more cautious about their health status. Apart from formal education, policymakers should also initiate awareness campaigns to diffuse health education to as many people as possible through the internet and other sources. Similarly, a dynamic and vibrant financial sector with a large number of financial institutions can provide necessary funds for developing health infrastructure even in far-flung areas. Therefore, the goal of financial development should also be assimilated into the nation's health policies. Results also suggested that policymakers in China should promote and encourage financial institutions in order to expand the utilization of financial services. Furthermore, financial investment should be increased in less developed areas in order to increase health services. Policymakers in China should focus on higher education and raise awareness among the masses about financial institutions that might raise their living standards and health outcomes. The affordability of financial resources might help in improving overall human development.

## Data Availability Statement

Publicly available datasets were analyzed in this study. This data can be found here: https://data.worldbank.org.

## Author Contributions

ZZ and RT: conceptualization, software, data curation, and writing-original draft preparation. MN: methodology, writing-reviewing, and editing. DK: visualization and investigation. All authors contributed to the article and approved the submitted version.

## Conflict of Interest

The authors declare that the research was conducted in the absence of any commercial or financial relationships that could be construed as a potential conflict of interest.

The article "Do Higher Education and Financial Institutions Improve Health in China? A New Perspective" was retracted in 2025. Reasons: an official misconduct investigation; compromised peer review; a compromised editor; unreliable results or conclusions.

## Publisher's Note

All claims expressed in this article are solely those of the authors and do not necessarily represent those of their affiliated organizations, or those of the publisher, the editors and the reviewers. Any product that may be evaluated in this article, or claim that may be made by its manufacturer, is not guaranteed or endorsed by the publisher.
